The article "Phospholipids containing ether-bound hydrocarbon-chains are essential for efficient phagocytosis and neutral lipids of the ester-type perturb development in Dictyostelium" was published in 2020. Journal: Biol Open.

# Phospholipids containing ether-bound hydrocarbon-chains are essential for efficient phagocytosis and neutral lipids of the ester-type perturb development in *Dictyostelium*

**DOI:** 10.1242/bio.052126

**Published:** 2020-07-16

**Authors:** Frederik Kappelt, Xiaoli Du Ma, Bassam Abou Hasna, Jessica M. Kornke, Markus Maniak

**Affiliations:** Zellbiologie, Universität Kassel, D-34109 Kassel, Germany

**Keywords:** Endoplasmic reticulum, Peroxisomes, Lipid droplets, GPAT, DHAPAT, Macropinocytosis

## Abstract

Lipids are the building blocks for cellular membranes; they provide signalling molecules for membrane dynamics and serve as energy stores. One path of their synthesis is initiated by glycerol-3-phosphate acyltransferase (GPAT), which in *Dictyostelium* resides on the endoplasmic reticulum. When an excess of fatty acids is present, it redistributes to storage organelles, the lipid droplets. Mutants, where the GPAT was eliminated by homologous recombination, produce fewer lipid droplets and are almost devoid of triacylglycerols (TAG), rendering them more resistant to cell death and cell loss in the developmental stages preceding fruiting body formation. The enzyme most closely related to GPAT is called FARAT, because it combines a fatty acyl-reductase (FAR) and an acyltransferase (AT) domain in its sequence. The protein is confined to the lumen of the peroxisome, where it transfers a fatty acid to dihydroxyacetone-phosphate initiating the synthesis of ether lipids, later completed at the endoplasmic reticulum. A mutant lacking FARAT produces lipid droplets that are devoid of the storage lipid monoalkyl-diacyl-glycerol (MDG), but the efficiency of spore formation in the developmental cycle is largely unaltered. Instead, these mutants are strongly impaired in phagocytosis of yeast particles, which is attributed to reduced synthesis of membrane phospholipids containing ether-linked chains.

## Abstract (precis)

**Summary:** Lean *Dictyostelium* mutants that fail to produce storage fat, survive starvation and succeed in spore formation, whereas cell strains impaired in ether-type membrane lipid production are perturbed in phagocytosis.

## INTRODUCTION

Membrane phospholipids not only act as a barrier between the cytoplasm of the cell and the extracellular space or the lumen of various organelles, but they also mediate cellular signalling. In particular this involves sphingolipids, the hydrolysis of phosphatidylcholine, and most of all, differential phosphorylation of the inositol head-group followed by local membrane recruitment of specific signalling proteins (Divecha and Irvine, 1995). Ground-breaking work on the last topic was conducted in the field of *Dictyostelium* (Parent et al., 1998; Iijima and Devreotes, 2002), although these lipid modifications were then shown to recruit cytoskeletal proteins to the sites of phagocytosis (Dormann et al., 2004) and turned out to be especially important for macropinocytosis (Hoeller et al., 2013; Kay et al., 2019; Vines and King, 2019) rather than chemotaxis (Hoeller and Kay, 2007).

The article "Phospholipids containing ether-bound hydrocarbon-chains are essential for efficient phagocytosis and neutral lipids of the ester-type perturb development in Dictyostelium" was published in 2020. Journal: Biol Open.

Similarly, neutral lipids not only serve as a reserve of energy and membrane building blocks but their storage organelle, the lipid droplet, fulfils an increasing number of unexpected physiological roles ranging from protein sequestration (Welte, 2015; Welte and Gould, 2017) to degradation (Moldavski et al., 2015). Across host cell kingdoms even various intracellular pathogens interact with lipid droplets (Barisch et al., 2015; Roingeard and Melo, 2017).

In *Dictyostelium*, lipid droplets (LDs) store neutral lipids mainly in the form of triacylglycerol (TAG) and, to a lesser extent, as monoalkyl-diacyl-glycerol (MDG) and steryl-esters (SE) (Du et al., 2013). In recent work, we have addressed the individual functions of the enzymes mediating the last step in TAG and MDG synthesis, DGAT1 and DGAT2 (Du et al., 2014). The latter enzyme plays a minor role in neutral lipid synthesis, as its knockout does not show a phenotype. On the contrary, DGAT1 is the main enzyme responsible for both TAG and MDG synthesis at the same time. Double knockout cells lacking both enzymes are severely affected in their ability to grow on bacteria as their natural food source (Du et al., 2014). They also become insensitive to the adverse effect of fatty acid addition, which in wild-type cells strongly perturbs the completion of development (Kornke and Maniak, 2017). In order to separate these pathways experimentally, and to be able to attribute individual phenotypes to either ether or ester lipids, we sought to interfere with the enzymes that initiate their pathways of synthesis.

Ester–lipid synthesis takes place in the endoplasmic reticulum and is initiated by the addition of a coenzyme A-activated fatty acid to the sn1-position of a glycerol-3-phosphate backbone. The enzyme forming this ester bond is called G-3-P acyltransferase (GPAT) (Takeuchi and Reue, 2009). The single *Dictyostelium* gene encodes an enzyme that localises to the endoplasmic reticulum (ER) and to LDs. A knockout mutant produces significantly reduced amounts of TAG when a fatty acid is present during their vegetative growth. Under these conditions, the mutants show increased phagocytosis and can successfully complete development, whereas wild-type cells are impaired in both processes.

In contrast, peroxisomes are the organelles where ether–lipid synthesis begins. In mammals, first an enzyme abbreviated DHAPAT adds a fatty acid to the sn1-position of dihydroxy-acetone-3-phosphate (Ofman et al., 1998). In a second step, this acyl-chain is then replaced by a fatty alcohol by ADPS (alkyl-dihydroxyacetone-phosphate-synthase) yielding the ether bond. Interestingly, the only crystal structure of this protein, which also allows to delineate the exact reaction mechanism, was derived from the *Dictyostelium* enzyme (Razeto et al., 2007).

The article "Phospholipids containing ether-bound hydrocarbon-chains are essential for efficient phagocytosis and neutral lipids of the ester-type perturb development in Dictyostelium" was published in 2020. Journal: Biol Open.

We have identified the acyltransferase mediating the first step described above. Because its sequence also bears a fatty acid reductase (FAR) domain N-terminal of the acyltransferase (AT), the protein was called FARAT. We show here, that FARAT indeed localises in peroxisomes, and mutants lacking this enzyme are unable to produce the storage lipid MDG. Probably, because many phosphatidylethanolamines as well as phosphoinositides in *Dictyostelium* are based on an ether–lipid backbone (Weeks and Herring, 1980; Clark et al., 2014), the mutants are strongly impaired in phagocytosis and show reduced macropinocytosis, as well as a rather mild developmental defect.

## RESULTS

### The initial step of TAG synthesis is carried out by GPAT on the ER and LDs

In mammalian cells, the majority of glycerolipid syntheses is initiated by GPAT enzymes of which four isoforms exist. GPAT1 and 2 are rather big enzymes of around 800 amino acids located in mitochondria. Their best homologue with only 26% identical residues in the *Dictyostelium* genome is DDB0305750, the gene that encodes FARAT (see below). A search with GPAT3 and 4, which are only around 450 amino acids in length, also turns up only a single gene, DDB0235400 (named *gpat*), with a better match of 44% identity to GPAT3 and 36% to GPAT4. The *Dictyostelium* GPAT protein comprises 488 residues and has a serine-rich region at the N-terminus, with 28 serines occurring within the 40 amino acids after the initial methionine and two predicted transmembrane domains followed by one acyltransferase domain (Fig. 1A). To analyse the subcellular localisation of GPAT, a GFP tag was either fused to the N-terminus of the protein or to its C-terminus. In the clone 1-8, GFP-GPAT shows a strong signal at the expected size of 83 kDa on a western blot, whereas the amount of GPAT-GFP is much lower (Fig. 1B), because in the latter clone (3-23) only about 20% of the cells appeared green by fluorescence microscopy. Nevertheless, both constructs yielded cells where a colocalization could be documented (Fig. 1C,D) between the GFP-tagged GPAT and the protein disulfide isomerase, a known ER-marker (Monnat et al., 1997). However, when the cells were provided with palmitic acid 3 h before fixation, so that they could accumulate lipid droplets, both GFP-GPAT and GPAT-GFP disappeared from the ER and were found to bind to the LD surface instead (Fig. 1E,F). This finding is consistent with our previous proteomic analysis of biochemically enriched LDs (Du et al., 2013).

The article "Phospholipids containing ether-bound hydrocarbon-chains are essential for efficient phagocytosis and neutral lipids of the ester-type perturb development in Dictyostelium" was published in 2020. Journal: Biol Open.

**Fig. 1.** **GPAT moves from the ER to lipid droplets.** (A) Schematic representation of the GPAT protein sequence drawn approximately to scale. The serine rich region (poly S) is represented by a blue box, followed by two predicted membrane domains (MD1 and 2, yellow). The acyl transferase (red) spans 125 amino acid residues. (B) Western blot detecting the two GFP fusions to the GPAT protein (green) in the region of 85 kDa as compared to the marker (M), with clone 1-8 expressing GFP-GPAT and double the number of cells from clone 3-23 producing the slightly smaller GPAT-GFP protein. The wild type (AX2) shows immunoreactivity to the severin (SEV) loading control. All strips originate from the same protein gel and blotting membrane. (C–F) Single confocal planes through fixed cells expressing GPAT fused to GFP (green channel) at the N-terminal end (C,E) or carrying the GFP-tag at the C-terminus (D,F), which were incubated in control medium (C,D) or in the presence of palmitic acid (+PA in E,F). The endoplasmic reticulum was revealed by immunofluorescence staining with anti-PDI (red in C and D), whereas lipid droplets were stained by LD 540 (red in E and F). The overlay images (OL) of red and green channels carry a scale bar of 5 µm.

In order to generate a mutant lacking the GPAT protein, we cloned the genomic *gpat* locus and inserted a cassette conferring resistance to Blasticidin S into the first of 6 exons (Fig. 2A). After electroporating a linear DNA-fragment into AX2 wild-type cells, we screened individual clones for the occurrence of homologous recombination by PCR analysis and selected two lines (1-21 and 2-6) with independent integration events for further investigation (Fig. 2B,C). *gpat^–^* mutants fed with a fluorescent fatty acid were found to contain only a few lipid droplets (Fig. 2D). Consistent with this observation, enzymatic tests (Fig. 2E) as well lipid extracts analysed by thin layer chromatography (Fig. 2F) and densitometry of (*n*=3 extractions) revealed that *gpat^–^* mutants produced about 70% less TAG but were largely unaffected in the level of MDG. To confirm that this phenotype originates from the disruption of the *gpat* gene, we transformed knockout strain 1-21 with either GFP-GPAT or GPAT-GFP expressing plasmids and documented the reappearance of wild-type levels of TAG again by enzymatic test (Fig. 2G) as well as by TLC (Fig. 2H).

The article "Phospholipids containing ether-bound hydrocarbon-chains are essential for efficient phagocytosis and neutral lipids of the ester-type perturb development in Dictyostelium" was published in 2020. Journal: Biol Open.

**Fig. 2.** **Lack of GPAT strongly affects TAG production.** (A) Diagram of the relevant region from the genomic *gpat* locus (upper line) with insertion of a Blasticidin S resistance cassette (lower line) by homologous recombination in the coding region of the first exon (E1). Binding sites for diagnostic primers are indicated by arrows and reside upstream or downstream of sequences used for targeting in the noncoding region (755) and in exon three (774) as well as in the BS-resistance gene (456). (B,C) PCR products from genomic DNA isolated from AX2 and two independently derived *gpat^−^* mutants (1-21 and 2-6). (B) Combining one primer binding 5′ upstream of the *gpat* coding region (775) and one primer specific for the resistance cassette (456), the disrupted copy of the *gpat* gene (*) can only be amplified in the mutants but not in wild type. An unrelated gene, *thioredoxin* (*trx*) was included to demonstrate the integrity of the template DNA. (C) Two primers situated in the *gpat* gene (775 and 774) amplify an 895 bp fragment from wild-type DNA, which increases to 2.5 kbp in the mutant strains, indicating the insertion of the BS^r^-cassette (gpat*) side by side with the presence of the original gene (*gpat*). The relevant sizes of the DNA marker (M) are given in base pairs. (D) Wild-type cells (AX2) and *gpat*-knockout strains (1-21 and 2-6) were cultivated in the presence of palmitic acid together with the lipid tracer C_1_-BODIPY-C_12_ for 3 h, fixed, and a single image plane was captured by confocal microscopy to reveal the lipid droplets. Scale bars: 5 µm. (E) Cells were stimulated by palmitic acid addition and allowed to form lipid droplets for 3 h. TAG-levels measured after 3 h through an enzymatic assay (see Materials and Methods). (F) Thin layer chromatography resolving steryl-esters (SE), monoalkyl-diacyl-glycerol (MDG) triacylglycerol (TAG), free fatty acids (FFA), cholesterol (CHL), as well as methyl-oleate (MO) as a loading control, from lipid extracts of AX2 and *gpat^−^* mutants incubated with palmitic acid aligned with the legend above. (G) Enzymatic assay of triglycerides and (H) TLC of neutral lipids from mutant 1-21 rescued by expression of GFP-GPAT (clone 1-12-6) or GPAT-GFP (clone 2-2) under conditions as used in panels E and F.

### Peroxisomal FARAT is responsible for MDG synthesis

As mentioned before, the other gene that appeared as a weak homologue of mammalian GPAT sequences was DDB0305750. Because its length of 1279 amino acids exceeded that of the other GPATs, we carried out a domain analysis and found a predicted FAR catalytic domain at the N-terminus, that is followed by the conserved AT centre and two blocks of nine or ten asparagine residues, which is not uncommon to *Dictyostelium* proteins (Malinovska et al., 2015). At its C-terminus the protein bears the tripeptide SKL, known as a peroxisomal targeting sequence type 1 (PTS1). The name FARAT was chosen for the protein and *fatA* indicates the corresponding gene (Fig. 3A). For localization studies, GFP was fused to the N-terminus of FARAT and could be detected as a band of 170 kDa on a western blot (Fig. 3B). Because a C-terminal fusion would have blocked the PTS1 signal, we inserted GFP just before the SKL sequence yielding the construct FARAT-GFP-SKL that was less efficiently produced in *Dictyostelium* cells (Fig. 3B). A full overlap of the GFP-tagged enzymes with RFP-labelled peroxisomes is documented in Fig. 3C and D. This distribution did not shift to lipid droplets (Fig. 3E,F), as seen for the human FAR1 protein (Exner et al., 2019) that corresponds to the N-terminal domain of *Dictyostelium* FARAT.

The article "Phospholipids containing ether-bound hydrocarbon-chains are essential for efficient phagocytosis and neutral lipids of the ester-type perturb development in Dictyostelium" was published in 2020. Journal: Biol Open.

**Fig. 3.** **FARAT is a strictly peroxisomal enzyme.** (A) Schematic drawing of the FARAT sequence approximately drawn to scale. The fatty acid reductase domain (FAR) is indicated by a green box, followed by the acyltransferase (AT, red), the poly N region (blue), and the C-terminal SKL tripeptide representing the type 1 peroxisomal targeting sequence. (B) Western blotting shows that a population of cells expressing N-terminally GFP (green) tagged FARAT (NP) shows a higher overall expression level than the population producing the C-terminally tagged enzyme (CP). In both cases some protein degradation, possibly occurring behind the poly-N region, is visible. AX2 does not show immunoreactivity in the region of 170 kDa as compared to the marker (M), but only to *Dictyostelium* vacuolin (VAC) used to illustrate equal loading of the gel. (C,D) Single confocal planes through fixed cells expressing FARAT fused to GFP (green channel) at the N-terminal end (C,E) or carrying the GFP-tag including a peroxisomal targeting sequence at the C-terminus (D,F). The peroxisomes were labelled by co-expression of RFP-SKL (red in C and D), whereas lipid droplets are stained by incorporation of the fluorescent fatty acid analogue C_1_-BODIPY-C_12_ (red in E and F). The size bar in the overlay images (OL) corresponds to 5 µm.

Homologous recombination with a genomic fragment of *fatA* (Fig. 4A) yielded two independently isolated strains (I/4 and II/22) that showed the insertion of a BS^r^-cassette into the *fatA* gene and correspondingly the absence of the wild-type copy (Fig. 4B,C). Although the mutants' LDs appeared to be normal by microscopy (Fig. 4D), thin layer chromatography revealed that the MDG band, previously identified by mass spectrometry (Du et al., 2014), was almost absent (Fig. 4E). Careful densitometry of three biological replicates revealed the residual amount of 13% MDG in the mutants (*P*<0.001). The amount of TAG, however, was not significantly different from the wild-type level (Fig. 4E); therefore, we refrained from conducting enzymatic TAG measurements. The *fatA*-knockout strain I/4 was chosen for further transformation to express either GFP-FARAT (clone I/17) or FARAT-GFP-SKL (clone I/3). Both constructs rescued the production of MDG to at least the same level as wild type (I/3) or even above AX2 levels (I/17), confirming that the gene disruption of *fatA* was indeed the cause for MDG loss (Fig. 4F).

The article "Phospholipids containing ether-bound hydrocarbon-chains are essential for efficient phagocytosis and neutral lipids of the ester-type perturb development in Dictyostelium" was published in 2020. Journal: Biol Open.

**Fig. 4.** **A *fatA* knockout is unable to synthesise neutral ether lipids.** (A) Sketch of the genomic *fatA* locus (upper line) with insertion of BS^r^ (lower line) by homologous recombination in the coding region of the first and second exon (E1, E2) upon which about 2.5 kb of the endogenous gene are lost. Binding sites for diagnostic primers are indicated by arrows and reside upstream or downstream of sequences used for targeting in the noncoding region (1198 and 1050) and in exon one (1118) as well as in the BS^r^-cassette (282). (B,C) PCR products from genomic DNA isolated from the wild-type strain (AX2) and two independently derived *fatA^−^* mutants (I/4 and II/22). (B) Combining one primer binding 5′ upstream of the *fatA* coding region (1198) and one primer specific for BS^r^ (282), the disrupted copy of the *fatA* gene (*) can only be amplified in the mutants but not in wild type. *Thioredoxin* (*trx*) was as a control for amplification. (C) One primer situated in exon 1 of the *fatA* gene (1118) and another oligonucleotide binding in its 3′ noncoding region (1050) amplify a 3332 bp fragment (*fatA*) from wild-type DNA, which decreases to 2.4 kbp in the mutant strains, indicating the insertion of the BS^r^-cassette (fatA*). The relevant sizes of the DNA marker (M) are given in base pairs. (D) Wild-type cells (AX2) and *fatA*-knockout strains (I/4 and II/22) were cultivated in the presence of palmitic acid together with the lipid tracer C_1_-BODIPY-C_12_ for 3 h, fixed, imaged by confocal microscopy. Scale bars: 5 µm. (E) TLC resolving neutral lipid classes as specified in Fig. 2F from AX2 wild-type cells and *fatA^−^* mutants I/4 and II/22 incubated with palmitic acid, as well as the rescue strains I/17 expressing GFP-FARAT and I/3 producing FARAT-GFP-SKL in the genetic background of the *fatA*-knockout I/4 (F).

### Interference with lipid synthesizing enzymes affects phagocytosis and development

Because cells lacking GPAT grew normally in liquid medium, we assumed that their ability to take up fluid by macropinocytosis was normal and resorted to measure phagocytosis. Using yeast particles as prey, both GPAT knockout lines were about 20% more efficient than wild-type cells (Fig. 5A). When the cells were pre-incubated with palmitic acid, so that they could accumulate lipid droplets, the overall efficiency of phagocytosis in wild-type cells decreased by 50%, as described before (Paschke et al., 2012), but *gpat* knockouts were not as dramatically affected, so that their performance remained 45% above wild-type levels (Fig. 5B).

The article "Phospholipids containing ether-bound hydrocarbon-chains are essential for efficient phagocytosis and neutral lipids of the ester-type perturb development in Dictyostelium" was published in 2020. Journal: Biol Open.

**Fig. 5.** **Lack of GPAT stimulates phagocytosis and protects from cell death in development.** (A) Quantitative measurement of particle internalization, shown as relative units [r.u.], in AX2 cells (closed circles) and *gpat*^−^ mutants (1-21, open squares and 2-6, open triangles). Data points are from three independent experiments ±s.d. and the curve connects the mean values. (B) Phagocytosis assays repeated in axenic medium containing palmitic acid (PA) for 3 h prior to measurement. (C) Cells expressing GFP or RFP were incubated for 3 h in growth medium containing (+PA) or lacking (−PA) palmitic acid and mixed with an equal number of cells of the other colour and allowed to develop on a moist agar surface. Bar diagram showing the percentage of wild-type (AX2, dark or light grey bars) and *gpat^−^* mutant (1-21, open bars) spores after harvesting. For bars 1 and 2, untreated cells were mixed in equal amounts and allowed to develop, whereas the wild type (dark grey) was subjected to a 3 h palmitic acid incubation (+PA) in bars 3 and 4. Conversely, the RFP producing *gpat^−^* mutant (open bar), and as a control the RFP-expressing wild type (light grey bar), were exposed to the fatty acid (+PA) in bars 5 and 6, while in the last combination (bars 7 and 8) all cells were grown in the presence of palmitic acid before undergoing development. Significance *P* is <0.0001 as indicated by four asterisks.

Because the ability to form lipid droplets also strongly impairs cell survival during development (Kornke and Maniak, 2017), we transformed AX2 wild-type cells to express GFP, while *gpat^–^* mutants produced RFP, for tracking their efficiency to form spores in mixing experiments. The results were compared to 50/50 mixtures of red and green fluorescent wild-type cells (Fig. 5C). If the cells originated from normal growth medium, the *gpat^–^* mutant and wild type each contributed 50% of the spores (bar 2 in Fig. 5C), and the same was seen, as expected, from mixtures with only wild-type cells (bar 1 in Fig. 5C). The mutants also formed about 90% of the spores when mixed with palmitic acid-treated wild type (bar 4 in Fig. 5C). However, when the *gpat^–^* mutants were pre-incubated in palmitic acid-containing medium, they were able to form spores four times more efficiently than wild-type cells (bars 5 and 6 in Fig. 5C). Consistent with this observation, *gpat^–^* mutants also resisted the adverse effect of fatty acid treatment whereas most of the LD-containing wild-type cells were lost over the 24 h hours of development (bars 7 and 8 in Fig. 5C).

The article "Phospholipids containing ether-bound hydrocarbon-chains are essential for efficient phagocytosis and neutral lipids of the ester-type perturb development in Dictyostelium" was published in 2020. Journal: Biol Open.

Overall, the *gpat^–^* mutants exactly mimic the behaviour of strains bearing fewer lipid droplets because a fatty acid-activating enzyme, FcsA, or one or both DGAT enzymes were mutated (Kornke and Maniak, 2017). Because in these strains TAG and MDG are reduced proportionally, the *fatA^−^* mutant, that is specifically affected in MDG synthesis, while producing normal amounts of TAG (see Fig. 4E), was subjected to the same type of mixing experiment. As seen in Fig. 6A, *fatA*-knockout cells are unable to efficiently contribute to the spore population when they were allowed to form lipid droplet in advance (bar 6′) and they also do not dominate mixtures where both strains were pre-treated with palmitic acid (bar 8′). Thus, cells lacking the FARAT enzyme and the neutral lipid MDG almost behave like wild-type cells (compare to Fig. 5C), most likely because they have unaltered TAG-levels.

**Fig. 6.** ***fatA***-**knockout cells are unaffected in development, but deficient in endocytosis.** (A) Bar diagram showing the percentage of spores formed after palmitic acid pre-incubation in the vegetative phase or untreated controls from GFP-expressing AX2 (dark grey bars) and RFP-expressing *fatA^−^* mutant (I/4, open bars). For AX2/AX2 mixtures and further details compare Fig. 5C. (B) Intracellular accumulation of a fluid-phase marker was measured as relative units [r.u.]. AX2 cells are represented by filled circles and the *fatA*^−^ mutants (I/4, II/22) by open symbols. Bars indicate the s.d. of *n*=3 biological replicates. (C) Determination of macropinocytosis was performed as in panel B, except that cells were allowed to form LDs from palmitic acid (+PA) 3 h prior to the assay. (D) Uptake of yeast particles is defective in the *fatA*-knockout strains (I/4 and II/22, open symbols) as compared to AX2 (black filled circles). Re-expression of either GFP-FARAT (dark green squares) or FARAT-GFP-SKL (light green squares) in the mutant I/4 fully restores phagocytosis. (E) When cells could form lipid droplets by the induction with palmitic acid (+PA) the differences between AX2 and *fatA*^−^ mutants is maintained (black lines) but rescues by expression of GFP-tagged FARAT proteins (green lines) are less efficient. For description of symbols see above. (F) TLC analysis of phospholipids in AX2 and in *fatA*^−^ and *gpat^−^* mutants. Phosphatidylethanolamine (PE) Phosphatidylinositol (PI), Phosphatidylcholine (PC), Lysophosphatidylcholine (LPC), and Phosphatidylserine (PS) were mixed in appropriate amounts to generate the markers (M). Since all marker lipids contain ester-bonded acyl chains, the ether species of PE and PI (red arrowhead) migrate slightly above the standards. The blue arrowhead points to Lysophosphatidylethanolamine as identified by its Rf value and positive reaction to ninhydrine spraying.

The article "Phospholipids containing ether-bound hydrocarbon-chains are essential for efficient phagocytosis and neutral lipids of the ester-type perturb development in Dictyostelium" was published in 2020. Journal: Biol Open.

In contrast to *gpat^−^* mutants, cells lacking FARAT grew somewhat more slowly in axenic medium. This consistently observed phenotype (average generation time 13.9 h versus 11.5 h in AX2 cells, but *P*<0.1 for *n*=3) can be at least in part attributed to a mild, but non-significant, reduction in the ability to take up fluid by macropinocytosis (Fig. 6B,C), however, a much stronger reduction was seen when phagocytosis was assayed (Fig. 6D). The addition of palmitic acid prior to the measurement neither influenced the relative fluid uptake (Fig. 6C) nor particle internalisation (Fig. 6E) of mutants versus wild type, although it depressed overall phagocytosis efficiency by about 50% (Paschke et al., 2012). Endocytic processes that are accompanied by dramatic morphological changes in the plasma membrane must strongly depend on the phospholipid composition. Therefore, we repeated TLC analysis of our mutants, now focussing on phospholipids. Though the global pattern of the *fatA^−^* mutant looked very similar to the wild type, a quantitative reduction was seen in the bands corresponding to PE and PI (Fig. 6F) being lipids that were previously identified to contain ether linked hydrocarbon chains (Weeks and Herring, 1980; Clark et al., 2014). The levels of these two phospholipids returned to normal upon expression of FARAT-GFP-SKL in the *fatA^−^* background, and it is notable that the defect in phagocytosis was concomitantly rescued (see Fig. 6D,E). Further inspection of the phospholipid pattern shows that none of the lipids detected in wild-type cells is missing in the *gpat^−^* mutant, it rather appears that the bands corresponding to PE, PI and, more clearly lysophospholipids, are becoming more intense, suggesting that from these species more ether variants are produced (Fig. 6F). Interestingly, the increased phospholipid levels in the *gpat^–^* mutants correlate with increased phagocytosis efficiency (see Fig. 5A,B).

## DISCUSSION

### *Dictyostelium* GPAT initiates TAG synthesis that interferes with the developmental program

Yeast has two enzymes with GPAT activity: Gat1p, which is localised in the ER-membrane and on LDs (Athenstaedt and Daum, 1997; Grillitsch et al., 2011), as well as Gat2p, which is confined to the ER (Athenstaedt and Daum, 1997; Zheng and Zou, 2001). The single *gat2* mutant produces 50% less TAG, whereas the *gat1* mutant produces about 40% more TAG (Zaremberg and McMaster, 2002). Thus, the single *Dictyostelium* GPAT localises like Gat1p (Figs 1 and 7) while the knockout resembles the effect of a yeast strain lacking Gat2p (Fig. 2E,F). In mammals, four GPAT activities were discovered. GPAT1 and 2 are related in size and sequence, and both localise to the mitochondrial outer membrane. The other pair of GPATs, isoforms 3 and 4, are ER enzymes (Cao et al., 2006), with GPAT4 able to move on to lipid droplets (Wilfling et al., 2013), similar to what we see for the *Dictyostelium* GPAT enzyme (Figs 1 and 7).

The article "Phospholipids containing ether-bound hydrocarbon-chains are essential for efficient phagocytosis and neutral lipids of the ester-type perturb development in Dictyostelium" was published in 2020. Journal: Biol Open.

**Fig. 7.** **Flow of proteins and lipids between organelles.** Schematic view of cellular organelles outlined by membrane monolayers (lipid droplets) or bilayers (ER, peroxisomes) in blue. Membrane proteins (red boxes) are inserted into the ER membrane and remain there, if they span the bilayer (DGAT1) or can move to the lipid droplet if only held by the lipid monolayer facing the cytoplasm (GPAT). FARAT (red dot) is a soluble protein that is post-translationally transported into the lumen of the peroxisome by virtue of its C-terminal type1 targeting sequence. Although its N-terminal domain is equivalent to the human FAR1 enzyme, *Dictyostelium* FARAT does not move from peroxisomes to the lipid droplet surface (broken red arrow). Lipid synthesis (black) is initiated in the ER membrane starting from glycerol -3-phosphate (G-3P) and acyl-coenzyme A (Ac-CoA, left). These substrates are converted by the action of GPAT to monoacylglycerol-3 phosphate (MAcG-3P, aka lysophosphatidic acid). Addition of the second acyl-chain yields diacylglycerol-3-phosphate (DAcG-3P, aka phosphatidic acid) which then is dephosphorylated to diacylglycerol (DAG) before the third acyl-moiety is linked by DGAT1 to generate triacylglycerol (TAG). Following a similar itinerary, ether lipid synthesis begins with the FARAT-catalysed bond formation between dihydroxyacetone-phosphate DHAP and Ac-CoA in the peroxisome (right). The acyl chain on DHAP is subsequently replaced by a long chain alcohol, formed by a reduction reaction on FARAT. This replacement reaction and another subsequent reduction of DHAP to G-3P are not shown, but together they yield monoalkylglycerol-3-phosphate (MAlG-3P) that is transferred to the ER. There one more acyl-chain is added, producing monoalkyl-monoacylglycerol-3-phosphate (MAlMAcG-3P), which, after removal of the phosphate-group (MAlMAcG), receives another acyl-moiety from DGAT1 to result in monoalkyl-diacylglycerol (MDG). Phospholipids carrying the more common ester bonds (PL), as well as ether-bonded variants (Eth-PL) are derived from various intermediates of the pathway.

The article "Phospholipids containing ether-bound hydrocarbon-chains are essential for efficient phagocytosis and neutral lipids of the ester-type perturb development in Dictyostelium" was published in 2020. Journal: Biol Open.

It is largely assumed that a common pathway exists for making phospholipids and neutral lipids [(Takeuchi and Reue, 2009) and references therein, Fig. 7]. Therefore, it may come as a surprise that the single GPAT enzyme detected in *Dictyostelium* appears to produce only storage lipids, not phospholipids, because the *gpat^–^* mutant shows a strong reduction in the TAG level (Fig. 2E,F), but in contrast some increase in phospholipids (Fig. 6F), suggesting that unused building blocks are rerouted into the latter pathway. Similarly, single *GPAT ^−/−^* mutant mice affecting isoforms 1, 3 and 4 show reduced fat content with some variation for tissues and organs (Hammond et al., 2002; Vergnes et al., 2006; Cao et al., 2014), while overexpression of GPATs 1, 2 and 3 leads to increased fat production (Igal et al., 2001; Cao et al., 2006; Wang et al., 2007). Also, only a few genetic manipulations in mammalian cells show an effect on the phospholipid composition, like the lack of GPAT1 (Lewin et al., 2008), or GPAT4 overexpression (Chen et al., 2008; Nagle et al., 2008). Whereas one can always infer redundancy between the GPATs to explain this observation, one additional problem is that some of the acyltransferases were initially mis-assigned. Chen et al. (2008) have clarified that earlier work on AGPAT6 (Beigneux et al., 2006; Vergnes et al., 2006) was really done on mice lacking the enzyme now known as GPAT4, and a similar confusion occurred when GPAT3 (Cao et al., 2006) was found to be identical to AGPAT10 (Sukumaran et al., 2009). Therefore, it is well possible that the mammalian GPAT family may gain new members when other putative AGPATS become analysed more rigorously. Along the same lines, it is also conceivable that one of the several as yet uncharacterised acyltransferases in the *Dictyostelium* genome is specifically responsible for the synthesis of phospholipids (Fig. 7).

Interestingly, some mammalian GPAT enzymes have cellular functions outside the main fat metabolizing tissues like liver, or fat storage organs like brown or white adipocytes: GPAT4 deficient mice specifically lack the ability to produce milk for feeding their pups (Beigneux et al., 2006), while GPAT2 plays a major role in spermatogenesis (Garcia-Fabiani et al., 2017). Stimulation of macrophages via toll-like receptors shifts metabolism to lipid storage in preparation to fight infection with concomitant increase of a set of lead enzymes, among them GPAT3 (Feingold et al., 2012). Moreover, efficient phagocytosis depends on lipolysis (Chandak et al., 2010). Thus, it is well conceivable that mammalian macrophages lacking GPAT3 or GPAT4 show compromised phagocytosis (Quiroga et al., 2019). In *Dictyostelium*, however, phagocytosis does not seem to depend on a TAG reservoir, because in *gpat^−^* mutants phagocytosis is even increased, whether or not the cells are challenged with palmitic acid (Fig. 5A,B).

The article "Phospholipids containing ether-bound hydrocarbon-chains are essential for efficient phagocytosis and neutral lipids of the ester-type perturb development in Dictyostelium" was published in 2020. Journal: Biol Open.

Instead, the dominant feature of *Dictyostelium* cells lacking GPAT is the resistance against fatty acid addition before development and the ability to efficiently produce spores under this condition (Fig. 5C). This supports previous observations on FcsA and the DGAT proteins (Kornke and Maniak, 2017) and means that the ability to make neutral lipids constitutes a risk for development. Because DGAT1 mutants lacked both TAG and MDG (Du et al., 2014; Kornke and Maniak, 2017), whereas in the *gpat^–^* mutants only TAG levels are reduced, while MDG is unaffected, we can now ascribe this perturbing effect specifically to excessive TAG storage, or ‘amoeboid obesity’.

### *Dictyostelium* FARAT produces neutral lipids and phospholipids essential for endocytosis

In yeast, both Gat enzymes forming the ester bond between glycerol-3-P also accept DHAP as a substrate, meaning that the synthesis of ether and ester lipids are not spatially separated in the cell (Zheng and Zou, 2001). In contrast, the Dictyostelium FARAT protein is found in peroxisomes (Figs 3C,D and 7) as also seen for the mammalian DHAP-acyltransferase (DHAPAT) (Liu et al., 2005). From here it does not move to the surface of lipid droplets (Figs 3E,F and 7) by virtue of its FAR domain, as shown for the human FAR1 protein (Exner et al., 2019). Not much work on DHAPAT has been done in mice (Rodemer et al., 2003), apparently because human patients lacking DHAPAT activity were found among the group carrying peroxisomal biogenesis disorders already 20 years ago (Ofman et al., 1998). The associated disease is called rhizomelic chondrodysplasia punctata type 2 and patients are characterised by shortening of the upper extremities, dysmorphic facial features, severe growth and mental retardation, where the last phenotype is ascribed to abnormal formation of myelin, which strongly depends on ether lipid synthesis (Sztriha et al., 2000).

DHAPAT enzymes from *Leishmania* (Al-Ani et al., 2011) and *Trypanosoma* (Zufferey et al., 2017) are much larger than their mammalian counterparts because they contain an N-terminal extension of unknown function. Interestingly, the ciliate *Tetrahymena* encodes the same bifunctional FARAT protein (Dittrich-Domergue et al., 2014) as *Dictyostelium*, where the N-terminal extension encodes a functional fatty acid reductase domain (Dittrich-Domergue et al., 2014) that may provide the fatty alcohol for the subsequent step in ether lipid synthesis (Fig. 7), catalysed by ADPS (Razeto et al., 2007). Whereas functional experiments on the *Tetrahymena* enzyme had to be performed in yeast (Dittrich-Domergue et al., 2014), the loss of DHAPAT in *Trypanosomes* appears to be lethal, but in a conditional mutant all ether lipid species decline, with a concomitant increase on ester phospholipids (Zufferey et al., 2017). The *Dictyostelium fatA^–^* mutant is almost devoid of the neutral lipid MDG, and residual amounts are assumed to originate from one of the surprisingly many polyketide synthases encoded in the genome (Zucko et al., 2007). Interestingly, DGAT1 accepts long-chain alcohols as substrates in wax-ester production and it is also instrumental in MDG biogenesis (Du et al., 2014). In addition, *fatA^–^* mutants also show a clear reduction in phospholipids (Fig. 6F) but remains viable, albeit growing somewhat more slowly. Its dominant phenotype is a dramatically reduced ability to take up particles by phagocytosis and a mildly affected macropinocytosis (Fig. 6B–E).

The article "Phospholipids containing ether-bound hydrocarbon-chains are essential for efficient phagocytosis and neutral lipids of the ester-type perturb development in Dictyostelium" was published in 2020. Journal: Biol Open.

Phagocytosis and macropinocytosis are similar processes in that a relatively large volume of extracellular space containing a particle or fluid, respectively, is internalised. This depends on the actin cytoskeleton and on associated proteins (e.g. coronin; Maniak et al., 1995; Hacker et al., 1997) in the same fashion. The same plasma membrane proteins are present or selectively excluded from nascent phagosomes and macropinosomes (Mercanti et al., 2006). The sequential appearance of the inositol lipids PI(3,4,5)P3 and PI(3,4)P2 has been followed with a time resolution of seconds and was found to be the same (Dormann et al., 2004). In support of this finding, knockout of the Dd5P4 phosphatase, the enzyme that performs the conversion of the above PIPs, perturbs phagocytosis and macropinocytosis to a similar extent (Loovers et al., 2007). On the other hand, individual knockouts of PI3 kinases (PIK1/2 double and PIK4 single) have been discovered and independently confirmed to affect macropinocytosis and phagocytosis differentially. (Zhou et al., 1995, 1998; Buczynski et al., 1997; Hoeller et al., 2013). Where the differences come from, is not finally established, but it might be due to different vesicle sizes as explained in Bloomfield et al. (2015).

In general, it appears that less inositol and ethanolamine type phospholipids lead to reduced endocytosis as seen for the *fatA^–^* mutant (Fig. 6B–E). Of course, this conclusion has to be taken with a grain of salt because for one, we cannot tell to which of the organelles or the plasma membrane these lipids are preferentially delivered, and secondly, within the scope of this paper, we cannot interfere with the production of only one of the PI and PE lipids individually. A conditional inositol mutant has been made very recently (Frej et al., 2016). It shows many changes in PI lipids, but most significant is the decrease in PIP2. Up to now, only slow growth in liquid medium and failure to produce plaques on bacterial lawn were reported, but the cells were not tested for macropinocytosis and phagocytosis with specific assays. Thus, future investigations should go into the function of the ethanolamine head-group in order to dissect the relative roles of phospholipids in endocytosis, especially since PE-ether lipids were recently demonstrated to have a strong impact on *Caenorhabditis* physiology (Shi et al., 2016). Finally, disregarding the head-group properties, ether-based phospholipids have strong impact on membrane structure and dynamics (Dean and Lodhi, 2018), and most notably affect professional phagocytes, where ether lipids are a truly vital component of neutrophils (Lodhi et al., 2015) and their remodelling specifically accompanies differentiation from the circulating monocyte to the macrophage (Wallner et al., 2014). In contrast, the inverse effect of increased phagocytosis (Fig. 5A,B) as observed in the *gpat^–^* mutants, may be due to higher levels of lysophospholipids (Fig. 6F), as demonstrated in mammalian macrophages (Ngwenya and Yamamoto, 1985; Balestrieri et al., 2009; Rubio et al., 2015).

The article "Phospholipids containing ether-bound hydrocarbon-chains are essential for efficient phagocytosis and neutral lipids of the ester-type perturb development in Dictyostelium" was published in 2020. Journal: Biol Open.

## MATERIALS AND METHODS

### Cell growth, mixing and development

Cells of the *Dictyostelium* AX2 strain ‘Gerisch’ (referred to as wild type) and mutants constructed in this genetic background were grown at 21°C in HL5+ medium (Formedium, UK) in shaking suspension and lipid droplet formation was induced by adding palmitic acid to a final concentration of 200 µM as described before (Du et al., 2013). For measuring competition during development, our published protocol and method of data evaluation (Kornke and Maniak, 2017) was followed, where the individual strains were labelled by expression of cytoplasmic GFP or RFP from pDNeo-2a based vectors (Dubin and Nellen, 2010). Each mixing experiment was conducted three times and over 100 spores each were counted. Between 1 and 4% of spores were non-fluorescent and thus omitted from the graphs. Endocytosis of TRITC-labelled yeast or TRITC-dextran was quantified as detailed in Rivero and Maniak (2006).

The article "Phospholipids containing ether-bound hydrocarbon-chains are essential for efficient phagocytosis and neutral lipids of the ester-type perturb development in Dictyostelium" was published in 2020. Journal: Biol Open.

### Molecular biology

DNA and protein sequences for *Dictyostelium gpat* (DDB0235400) encoding GPAT and *fatA* (DDB0305750) encoding FARAT were obtained from the fully sequenced genome (Eichinger et al., 2005) via http://dictybase.org where they are also linked to studies of expressed sequence tags. Transmembrane regions and targeting signals were identified at http://ch.EMBnet.org.

To fuse GPAT with GFP, reverse transcribed total mRNA from *Dictyostelium* was used as a template, primers 771 (CCGGATCCAAAATGGGGAAAGAAAGTAGTGATAATTCATCATTATCG) and 772 (CCGGATCCTTATTCGTTTGGGGTTGCCAATTTTC) further amplified the complete coding sequence of the *gpat* gene, now flanked by BamHI restriction sites. This fragment was inserted into the unique BamHI site of plasmid 68 pDNeoGFP (Jenne et al., 1998) generating vector 937 that expresses GFP-GPAT in clone 1-8. The opposite construct, GPAT-GFP (plasmid 938) produced by clone 3-23, was produced similarly, except that primer 771 was combined with primer 773 (CCGGATCCTTCGTTTGGGGTTGCCAATTTTC) which eliminated the stop-codon, so that translation could proceed into the GFP coding region provided by plasmid 48 pDd-A15-GFP w/o ATG [(Gerisch et al., 1995) as modified by Hanakam et al. (1996)].

To amplify *fatA* from cDNA primers 1023 (ATGGTAGTATTAGCAAATTTTTATGCTGGTAAAAC) and 1024 (TTAAAGTTTTGAAGATAATAATGGGAAATCTTCAAC) were used. The cDNA copy was ligated into pGemT-easy (Promega) resulting in plasmid 1210. This plasmid was taken as a template for a second amplification with primers 1167 (GTCGACAAAAATGGTAGTATTAGCAAATTTTTATG) and 1168 (CTCGAGTTAAAGTTTTGAAGATAATAATGGGAAATC) to provide the gene with SalI and XhoI restriction sites. Again, the amplicon was ligated into pGemT-easy yielding plasmid 1325. Subsequently the gene was inserted via SalI and XhoI into pDNeo2a-GFP (Dubin and Nellen, 2010) resulting in a GFP-FARAT expressing construct (Plasmid 1326).

To tag the FARAT protein on its C-terminal end, a PTS1 (peroxisomal targeting sequence type 1) was first fused to the C-terminus of the GFP in pDNeo2a-GFP to prevent a mis-localisation of FARAT. Therefore, primers 1101 (AGATCTAAATTATAACTCGAGCTCGGGTC) and 1103 (GTTATAATTTAGATCTTGTCGACCCTTTGTATAGTTC) were used to amplify the whole plasmid and to add the PTS1 by PCR resulting in Plasmid 1271 (pDneo2a-GFP-PTS1). Primers 1106 (CTTCTGCAGAAAATGGTAGTATTAGCAAATTTTTATG) and 1107 (GAAGGATCCAGATAATAATGGGAAATCTTC) were used not only to add PstI and BamHI restriction sites to *fatA*, but also to delete the endogenous PTS1 signal and the stop codon. The amplicon was ligated into pGemT-easy for sequencing and subsequently cloned into plasmid 1271, resulting in plasmid 1273 that expresses FARAT-GFP-PTS1 in two Dictyostelium clones, I/3 and I/8.

The article "Phospholipids containing ether-bound hydrocarbon-chains are essential for efficient phagocytosis and neutral lipids of the ester-type perturb development in Dictyostelium" was published in 2020. Journal: Biol Open.

To disrupt the *gpat* gene by homologous recombination, the gene was amplified from *Dictyostelium* genomic DNA using primers 771 and 774 (CCGGATCCCCAACTATTAAACAAGTTAGTCTTAATGG) and the product was maintained in pGemT-easy (Promega) as vector 922. Next, this vector was transformed into a *Dam**^−^** Escherichia coli* strain so that the ClaI restriction site in the first exon could be cut, the overhangs were filled in with Klenow polymerase and the SmaI-flanked BS^r^ cassette from pLPBLP (Faix et al., 2004) was integrated. The product, in which the cassette was transcribed in opposite direction with respect to *gpat*, was numbered 931. Digestion with EcoRI and NotI produced a fragment that was electroporated into *Dictyostelium*. The resulting clones were screened by PCR on their genomic DNA using a primer 775 (CATATAGCAATAGAATCAAGTTTGATAAAAATAC), that was not part of the targeting construct, in combination with either primer 456 (GGAGTTGATTTCAGACTATGC), binding within the resistance gene or, alternatively, primer 774. Clones 1-21 and 2-6, derived from two independent transformation events, were further investigated in this work.

For the insertion of a BS^r^-cassette into the *FatA* gene, Plasmid 1210 was digested with SwaI and EcoRV so that a 2.5 kb region of the *fatA* was deleted. Then a SmaI cut BS^r^ cassette from pLPBLP was ligated in between the two remaining flanking sites of *fatA* of approximately 700 bp. The resulting plasmid 1245 contains the 1.5 kb BS^r^-cassette in the same orientation as *fatA*. The construct was digested with EcoRI before electroporation to facilitate homologous recombination. Primers 1118 (GCTATCACCGAACGTATCCTCG) and 1050 (CAAATGCTTGGGGGATTTTAG) were used to confirm the correct integration of the BS^r^ cassette. 1118 binds within exon 1 and 1050 hybridises downstream of *fatA,* in a position that was not part of the electroporated fragment. To analyse the correct upstream integration, primers 1198 (CAATGTTGCCCTTAAGTTAAGAGTC) and 282 (CCAACCCAAGTTTTTTTAAACC) were used. The former is targeted to a position upstream of *fatA*, whereas primer 282 binds in the Blasticidin S resistance cassette. Knockout clones I/4 and II/22 were obtained from two independent electroporation events.

### Lipid analysis

The classical method of lipid preparation by Bligh and Dyer (1959) was adapted as described previously (Du et al., 2013). Subsequently, neutral lipids from three independent experiments were separated by thin-layer chromatography (TLC) on silica plates using two solvents. When the first solvent front (hexane:diethylether:acetic acid 80:20:1) had reached two-thirds of the separation distance, the plate was air dried and further developed in a second solvent system (hexane:diethylether 49:1) to completion. To visualise the lipids, TLC plates were stained for 3 s with copper sulfate (0.6 M in 8.5% phosphoric acid) and heated to 160°C for 15 min to conduct the charring reaction. For phospholipid separation, we used high performance TLC (HPTLC) plates with a silicagel S 60 Nano-ADAMANT surface (Machery-Nagel, Ref. 821140). The separation procedure is detailed in (Leray et al., 1987). Briefly, HPTLC plates were impregnated with 2.3% Boric acid dissolved in ethanol allowed to dry under a fume hood for 5 min and further treated for 15 min at 100°C in a hot-air oven. The bottom of the TLC chamber was filled with a solvent system containing chloroform/ethanol/water/triethylamine (30/35/7/35v/v) and the sides were decorated with filter paper to provide a homogeneous atmosphere. After lipid spotting, the HPTLC plate was placed in the chamber and developed until the solvent reached the top of the plate. After drying, the plate was dipped into a solution containing 0.16 M NaOH, 0.06 M HCl and 1 g l^−1^ 8-Anilino-1-naphtalene-sulfonic acid (Sigma-Aldrich, ref. A1028), air-dried, and visualised under UV-light. Phospholipids were identified by co-migration with the following standards: Phosphatidylinositol (Sigma-Aldrich, 79403), L-A-Phosphatidylserine (Sigma-Aldrich, P7769), Lyso-Phosphatidylcholine (Avanti Lipids, 830071P), 1,2-dioleoyl-sn-glycero-3-phosphocholine (Avanti Lipids, 850375P) and 1,2-dioleoyl-sn-glycero-3-phosphoethanolamine (Avanti Lipids, 850725P). In addition, cellular triacylglycerol amounts were quantified by a coupled enzymatic reaction described previously (Du et al., 2013) in three biological replicates and displayed with mean±s.d. shown in the bar diagram. The values of unstimulated cells were subtracted and the AX2 wild type was used as a reference (for reasons see Du et al., 2014).

The article "Phospholipids containing ether-bound hydrocarbon-chains are essential for efficient phagocytosis and neutral lipids of the ester-type perturb development in Dictyostelium" was published in 2020. Journal: Biol Open.

### Immunofluorescence experiments, GFP microscopy and western blotting

Immunofluorescence experiments, GFP microscopy and western blotting were performed as described before (Maniak et al., 1995). The distribution of the endoplasmic reticulum was shown by indirect immunofluorescence using undiluted mouse monoclonal antibody supernatant raised against the protein-disulfide isomerase (PDI, MAb 221-64-1) (Monnat et al., 1997). Monoclonal antibodies were detected using CY3-coupled goat-anti-mouse polyclonal secondary antibodies (Dianova). The lipid droplet-specific dye LD540 (Spandl et al., 2009) was diluted from its stock (0.5 mg ml^−1^ in ethanol) to a final concentration of 0.3 µg ml^−1^ in phosphate-buffered saline (PBS) and used to stain fixed cells for 30 min instead of using an antibody. Alternatively, LDs were metabolically labelled with the fluorescent fatty acid analogue C_1_-BODIPY-C_12_ (5 µM final concentration, Thermo Fisher Scientific) supplemented together with palmitic acid for 3 h in growth medium. Peroxisomes were labelled by co-expression of RFP-SKL (Schmauch and Maniak, 2008). Images were taken as single confocal planes using a Leica TCS-SP laser scanning microscope. In western blots, mouse monoclonal antibody 264-449-2 (available from Millipore) was used to detect GFP, whereas antibodies directed against *Dictyostelium* severin (42-65-11; Schleicher et al., 1984) and vacuolin (263-79-2; Wienke et al., 2006) served as loading controls.
